The article "Effects of the Ultrasound-Guided Stellate Ganglion Block on Hemodynamics, Stress Response, and Gastrointestinal Function in Postoperative Patients with Colorectal Cancer" was retracted in 2023. Reasons: unreliable results or conclusions; lack of ethics approval or compliance; concerns about the data; concerns about the peer review.

# Effects of the Ultrasound-Guided Stellate Ganglion Block on Hemodynamics, Stress Response, and Gastrointestinal Function in Postoperative Patients with Colorectal Cancer

**DOI:** 10.1155/2022/2056969

**Published:** 2022-07-14

**Authors:** An Xie, Xianjie Zhang, Feng Ju, Wen Li, Yukai Zhou, Dan Wu

**Affiliations:** ^1^Department of Anesthesiology, People's Hospital of Deyang City, Deyang, Sichuan 618000, China; ^2^People's Hospital of Deyang City, No. 173 Taishan Road, Deyang, Sichuan Province, China

## Abstract

**Objective:**

The aim of the study was to study the effects of the ultrasound-guided stellate ganglion block on hemodynamics, stressful response, and postoperative gastrointestinal functions in patients with colorectal cancer.

**Methods:**

A total of 100 patients with colorectal cancer hospitalized from January 2021 to December 2021 were selected. After anesthesia induction, the right stellate ganglion block was performed under ultrasound guidance in the research group and the general anesthesia was performed in the control group. The heart rate (HR), mean arterial pressure (MAP), epinephrine, cortisol, self-rating anxiety scale (SAS), Ramsay sedation score (RSS), postoperative bowel sound recovery time, anal exhaust time, and the incidence of gastrointestinal adverse reactions 24 hours after operation were studied pre-and post-24-hour anesthesia induction.

**Results:**

Following 24-hour operation, the HR and MAP values were largely reduced (*p* < 0.05). Following 24-hour operation, epinephrine and cortisol became obviously higher (*p* < 0.05). After 24-hour operation, the levels of epinephrine and cortisol in the research group were greatly lower. The score of the SAS in the study cohort was less than that of the controls (*p* < 0.05). The RSS of the research group was obviously increased (*p* < 0.05). The recovery time of intestinal sound and the anal exhaust time of the study cohort became remarkably shorter (*p* < 0.05). The incidence of gastrointestinal adverse reactions 24 hours after operation of the study cohort was much less common (*p* < 0.05).

**Conclusion:**

The ultrasound-guided stellate ganglion block can reduce the fluctuation of blood circulation during radical resection of colorectal cancer, reduce postoperative gastrointestinal dysfunction and stress reaction, relieve patients' anxiety, and contribute to the recovery of gastrointestinal function.

## 1. Introduction

Colorectal cancer is a malignant disease with a high incidence. Most of the patients had no obvious symptoms in the early stage, and most of the patients are found in the middle and the late stage. Common clinical manifestations are usually changes in defecation habits, such as abdominal pain and diarrhea [1]. Among the global cancer diseases, the incidence of colorectal cancer is the third and the mortality rate is the second [2]. In 2015, there were 387600 new colorectal cancer patients in China, accounting for 9.87% of all new cancer patients. A total of 187100 patients died of colorectal cancer, accounting for 8.01% of all cancer patients [3]. From the global perspective, the incidence of colorectal cancer in the United States has been declining in the past decade, while the incidence and mortality of colorectal cancer in China have increased year by year [4–6]. Apparently, colorectal cancer has become a major public health problem that threatens health of residents around the world.

So far, the most important and effective treatment for colorectal cancer is surgical treatment [7, 8]. In addition, the disturbance is caused by operation in varying degrees [9, 10]. Long-term postoperative inhibitions probably cause an increase in the incidence of postoperative intestinal obstruction [11]. The severe cases can increase the risk of reoperation with systemic inflammatory response syndrome or multiple organ dysfunction syndromes [14, 15].

Previous studies have shown that the stellate ganglion block (SGB) can inhibit surgical stress and inflammation and adjust the level of gastrointestinal hormones in rats undergoing gastrointestinal surgery [16], so that the digestive function of rats undergoing gastrointestinal surgery can quickly return to normal [17, 18]. The stellate ganglion is a ganglion formed by the combination of the inferior cervical ganglion, and the first thoracic ganglion and receives the T1∼T2 nerve at the same time. Its branches can innervate the blood vessels, sweat glands, pilus muscle, bone, joints, and so on. The medial side of the stellate ganglion is the esophagus, trachea, recurrent laryngeal nerve, and long cervical muscle. The lateral side is the anterior scalenus muscle. The front is the carotid sheath, vertebral artery, and vertebral vein, and the rear is the cervical transverse process. It reversibly blocks the stellate ganglion and its adjacent sympathetic ganglia to block the preganglionic and postganglionic nerve fibers in the innervation area of these ganglia so that the disorder of autonomic nerve function can be relatively balanced. However, there are few studies on the stellate ganglion block and early recovery of gastrointestinal function in clinical work.

## 2. Materials and Methods

### 2.1. General Information

A total of 100 patients with colorectal cancer hospitalized from January 2021 to December 2021 were selected. A total of 100 patients with colorectal cancer were randomly divided into the study cohort and the control cohort, including 50 cases, respectively. In the research group, there were 25 males and 25 females, aged from 48 to 69 years old, with an average age of (58.36 ± 4.22) years. The body mass index was 18.5∼24.0 kg/m^2^, with an average BMI of (21.48 ± 2.33) kg/m^2^. In the control group, there were 24 males and 26 females, aged from 47 to 69 years, with an average age of (58.42 ± 4.17) years. The body mass index was 18.6∼24.0 kg/m^2^, with an average BMI of (21.51 ± 2.29) kg/m^2^.

Inclusion criteria were as follows: (1) patients who underwent colorectal cancer surgery within a limited period of time; (2) patients aged between 45 and 65 years old; (3) ASA grade I∼II; (4) cardiopulmonary function was basically normal, no obvious heart, liver, kidney, endocrine diseases, preoperative laboratory, and related imaging examination results were not significantly abnormal.

Exclusion criteria were as follows: (1) patients with a history of upper respiratory tract infection within 2 weeks; (2) those with an obvious abnormality of heart, liver, and renal function; (3) those with a history of drug and alcohol abuse; (4) those with a history of allergy to narcotic drugs; (5) long-term use of anticoagulant drugs; (6) those with skin injury or infection at the puncture point of the neck; (7) those with an abnormal immune system; (8) those who refused to participate in this study; (9) the clinical data were incomplete.

### 2.2. Methods

#### 2.2.1. Technical Route

As shown in Figure 1.

#### 2.2.2. Treatment Regimen

The patients visited the day before the operation and were asked about their relevant medical history. The patient and his family were informed about the anesthesia-related procedures and possible complications.

The control group received routine general anesthesia. After entering the room, the peripheral venous pathway was established. The electrocardiogram, heart rate, blood oxygen saturation, noninvasive arterial blood pressure, and EEG bispectral index were monitored by using the Drager Infinity C500 anesthesia monitor. All patients were given general anesthesia by endotracheal intubation. Anesthesia induction consisted of midazolam 0.03 mg/kg, fentanyl 3∼5 *μ*g·kg^−1^, propofol 1.5∼2.0 mg·kg^−1^, and cis atracurium 0.2 mg·kg^−1^. The patient's BIS was in the range of 45 to 55, the muscle was completely relaxed, and endotracheal intubation was performed using a visual laryngoscope. After successful intubation, mechanical ventilation was performed, and the tidal volume was 6∼8 ml·kg^−1^. The partial pressure of end-expiratory carbon dioxide was maintained at 35∼45 mmHg, and the respiratory rate was adjusted according to the partial pressure of end-expiratory carbon dioxide. Continuous intravenous infusion of propofol and remifentanil was used for sedation and analgesia during anesthesia maintenance. The maintenance dose was adjusted according to the BIS value, which should be maintained in the range of 50–60. For the fluctuation of hemodynamics during operation, under the condition of ensuring the appropriate depth of anesthesia, the blood pressure was maintained in the range of ±20% of the basic value. Above or below this range, urapidil or ephedrine can be administered to regulate blood pressure. When the blood pressure was reduced, fluid replacement treatment can be carried out according to the specific conditions. The heart rate would be maintained at 50∼100 beats/min. If it was higher or lower than this range, after excluding the causes of blood loss, arrhythmia, and improper depth of anesthesia, intravenous injection of esmolol or atropine can adjust the heart rate.

In the research group, the right stellate ganglion block was performed under ultrasound guidance after anesthesia induction. After induction of general anesthesia, the planetary ganglion was blocked at the level of the seventh cervical vertebra on the right under the guidance of ultrasound. The medical staff arranges the patient to lie down, turns the patient's head to the left, disinfects the puncture point, and spreads a surgical towel. After determining the structures of the thyroid, carotid artery, vertebral artery, inferior thyroid artery, trachea, and esophagus, the puncture needle was inserted from the lateral transverse plane of the probe, and the carotid sheath was pushed to the outside as far as possible. To avoid vascular damage, when the tip of the needle entered the deep side of the prevertebral fascia on the surface of the cervical longus muscle, 0.2% ropivacaine hydrochloride 4 ml is slowly injected after pumping no blood, gas, or cerebrospinal fluid.

Tropisetron was administered intravenously 30 minutes preoperation ending. The intravenous analgesia pump was routinely used in all patients after operation. The formula was fentanyl 10 *μ*g·kg^−1^+tropisetron 4 mg + dexmedetomidine 0.1 *μ*g·kg^−1^·h^−1^ diluted to 100 ml to relieve postoperative pain. After the patient entered the anesthesia recovery room, a suitable position for the patient was arranged. In addition to psychological support measures by using words such as comfort and encouragement, nurses needed to make use of nonverbal skills, such as guiding patients to communicate with patients by blinking, nodding, and shaking their heads. Mental health education was given after the patients were fully conscious. According to the patient's own tolerance, the nurse carried out massage nursing to the patient according to the standard of gentle operation.

#### 2.2.3. Observation Indicators

1. To study the heart rate (HR) and mean arterial pressure (MAP) before anesthesia induction and 24 hours after operation.
2. To study the levels of epinephrine and cortisol before and 24 hours after anesthesia induction, peripheral blood 5 ml was collected and centrifuged at 3000 for 5 minutes. The supernatant (plasma) was stored in a refrigerator at −80°C. The levels of adrenaline and cortisol were detected by using the ELISA kit. All ELISA kits are purchased from the CUSABIO company.
3. To study the scores of the self-rating anxiety scale (SAS) and the Ramsay sedation score (RSS) during anesthesia recovery, the score of the SAS was divided into 4 grades, including 20 items [19], of which, 15 items were described by negative words, calculated according to 1–4 scores. 5 items were described by positive words, calculated according to 4–1 scores. The anxiety score of each item was added to get a rough score. On this basis, the integer part of the number multiplied by 1.25 was the final anxiety score. According to the standard of the Chinese norm, if the score was ≥50, it was considered that the patient has anxiety disorder. The Ramsay sedation score scale was proposed by Ramsay in 1974 [20] and the Cronbach's *α* coefficient was 0.94. The score range of the scale was 1–6.
4. To study the recovery time of intestinal sound and the time of anal exhaust after operation.
5. To study the incidence of gastrointestinal adverse reactions 24 hours after operation.

### 2.3. Statistical Analysis

The statistical analyses of the results were carried out by SPSS 24.0. Statistical figures were plotted by Graphpad Prism 8.0. Data conforming to a normality distribution were represented as the mean ± standard deviation (±*s*). The paired samples *t*-test was employed for intragroup comparisons, and the independent sample *t*-test was used for inter-group comparisons. *p* < 0.05 was considered statistically significant.

## 3. Results

### 3.1. The HR and MAP Values Were Studied before and 24 Hours after Anesthesia Induction

Twenty-four hours after operation, the HR and MAP values in both groups were significantly lower than those before anesthesia induction (*p* < 0.05). See Tables 1 and 2.

### 3.2. The Levels of Epinephrine and Cortisol before and 24 Hours after Anesthesia Induction

Following 24-hour operation, the levels of epinephrine and cortisol in both groups were significantly higher than those before anesthesia induction (*p* < 0.05). Twenty-four hours after operation, the levels of epinephrine and cortisol in the research group were considerably lower than those in the control group (*p* < 0.05) ( see Tables 3 and 4).

### 3.3. The Score of the SAS Scale and the RSS Scale during the Recovery Period of Anesthesia

The score of the SAS in the study cohort was considerably less than that in the control group (*p* < 0.05). The RSS score of the research group was greatly higher (*p* < 0.05) ( see Table 5).

### 3.4. The Recovery Time of Intestinal Sound and the Time of Anal Exhaust after Operation

The recovery time of intestinal sound and the anal exhaust time in the study cohort became statistically shorter (*p* < 0.05) (see Table 6).

### 3.5. The Incidence of Gastrointestinal Adverse Reactions 24 Hours after Operation

The incidence of gastrointestinal adverse reactions 24 hours after operation in the research group was remarkably lower than that in the control group (*p* < 0.05) (see Table 7).

## 4. Discussion

Colorectal cancer is a malignant tumor of the digestive system, which is caused by genetic, environmental, and other factors. The global mortality rate of colorectal cancer is about 50%, with the fourth fatality rate [23]. The incidence of the disease is increasing in many countries because of their bad habits [24]. Nowadays, people's material life has improved significantly. These factors have led to the fastest increase in the incidence of colorectal cancer in China [25]. The main treatment for patients with early colorectal cancer is surgery, while patients with advanced colorectal cancer are treated with surgery on the basis of preoperative radiotherapy and chemotherapy [26]. However, operation and anesthesia can cause stress and inflammatory reactions and prolong the time needed for gastrointestinal recovery after operation [27, 28].

The sympathetic nervous system is widely distributed in the palace of primary and secondary lymphoid organs. The adrenergic receptors are also widely distributed in immune cells such as macrophages and neutrophils. When sympathetic excitation occurs, sympathetic postganglionic fibers release catecholamines to activate adrenergic receptors of immune cells in lymphoid organs [29, 30]. In addition, sympathetic excitation can inhibit parasympathetic excitability. Surgical stimulation increased sympathetic excitability, aggravated perioperative inflammatory reaction, and delayed the recovery time of postoperative gastrointestinal function [31]. Therefore, choosing appropriate anesthesia, maintaining appropriate intraoperative management measures, and taking appropriate intervention measures to prevent excessive excitation of the sympathetic nervous system are very important for patients to quickly recover gastrointestinal function for anesthesiologists.

The stellate ganglion is a kind of a sympathetic ganglion. Its fibers can widely dominate the skin of the heart, brain, throat, shoulder and neck, trachea and bronchus, lung, and chest wall [32]. The stellate ganglion block refers to the injection of local anesthetic into the stellate ganglion and the loose connective tissue around it to inhibit the excitement of nerve cells by blocking the flow of sodium ions into the cell membrane. Reducing impulse transmission can achieve the purpose of reversibly blocking the stellate ganglion and its branches [33]. In recent years, ultrasound technology has become more and more mature and it has been widely used in all kinds of nerve block anesthesia. With the application of ultrasonic imaging technology in the process of the stellate ganglion block, we can observe the nerves, the blood vessels, the pleura, and other important tissues in real time and locate them accurately. We can also observe the specific location of the puncture needle and the distribution of anesthetics. By properly adjusting the puncture needle to make the drug spread evenly, we avoid an incomplete block and improve the success rate of puncture. Under the guidance of this visualization technique, we can use the minimum amount of anesthetic to achieve the best anesthetic effect and reduce the incidence of complications of the stellate ganglion block. Ultrasound has no radiation and will not cause damage to the human body during operation, which makes it more popular in clinics. Based on the advantages of ultrasound, the effects of the ultrasound-guided stellate ganglion block on hemodynamics and stressful response in patients with colorectal cancer were studied.

The results have proved that the ultrasound-guided stellate ganglion block can reduce the fluctuation of blood circulation, reduce the concentration of epinephrine and cortisol in peripheral blood, and reduce gastrointestinal dysfunction and stress reaction after operation. The anxiety can be relieved during the perianesthetic period so that the patients pass the anesthetic recovery period safely. This was mainly because all patients in this study underwent the ultrasound-guided stellate ganglion block by the same anesthesiologist. Some studies pointed out that the left stellate ganglion block can increase left ventricular diastolic pressure and myocardial oxygen consumption, weaken myocardial contractility, reduce the left ventricular ejection fraction, and increase the cardiac QT interval, while the right stellate ganglion block can effectively reduce sympathetic nerve activity, reduce cardiac oxygen consumption, and has little effect on circulatory fluctuation [34, 35]. In addition, the stellate ganglion block can regulate autonomic nerve function, inhibit hyper sympathetic nerve, dilate the diameter of central and peripheral blood vessels, weaken stress response in vivo, and maintain normal blood perfusion in tissues and organs of the whole body [36]. The stellate ganglion block can also prolong the atrial effective refractory period and increase cardiac electrophysiological stability [37], which indicates maintaining the stability of the circulatory system in patients. Moreover, the stellate ganglion block can inhibit abnormally active sympathetic activity, reduce the levels of catecholamine and cortisol, weaken the body's stress response, and promote the recovery of human immune function to further inhibit inflammation [38]. At the same time, it can improve the blood circulation of the hypothalamus [39] and make the patients pass through the recovery period safely. It has been found that the stellate ganglion block can inhibit oxidative stress and early inflammatory response in patients with hemorrhagic shock, inhibit hypothalamic sympathetic nerve excitation, improve local tissue ischemia and hypoxia, and shorten the intestinal peristalsis time and anal exhaust time [40]. There are some limitations in this study. First, the sample size of this study is not large and it is a single-center study, so bias is inevitable. In future research, we will carry out multicenter, large-sample prospective studies, or more valuable conclusions can be drawn.

In conclusion, the ultrasound-guided stellate ganglion block can reduce the fluctuation of blood circulation during radical resection of colorectal cancer, the concentration of epinephrine and cortisol in peripheral blood, and gastrointestinal dysfunction and stress reaction after operation. The anxiety can be relieved during the perianesthetic period to promote the recovery of gastrointestinal function after operation.

## Figures and Tables

**Figure 1:** Technology roadmap.

**Table 1:** Comparison of the HR before and 24 hours after anesthesia induction.

Group	Before induction of anesthesia (times/min)	24 hours after operation (times/min)
Control group (*n* = 50)	78.54 ± 7.19	73.82 ± 6.11^*∗*^
Research group (*n* = 50)	78.35 ± 7.12	71.69 ± 6.23^*∗*^
*t* value	0.133	1.726
*p* value	0.894	0.087

Note: the symbol^*∗*^represents the comparison of 24 hours before and 24 hours after anesthesia induction in this group, *p* < 0.05

**Table 2:** Comparison of the map value before and 24 hours after anesthesia induction.

Group	Before induction of anesthesia (mm Hg)	24 hours after operation (mm Hg)
Control group (*n* = 50)	95.19 ± 9.08	92.54 ± 9.19^*∗*^
Research group (*n* = 50)	95.24 ± 9.02	91.38 ± 9.12^*∗*^
*t* value	0.028	0.634
*p* value	0.978	0.528

Note: the symbol^*∗*^represents the comparison of 24 hours before and 24 hours after anesthesia induction in this group (*p* < 0.05).

**Table 3:** Comparison of the epinephrine levels before and 24 hours after anesthesia induction.

Group	Before induction of anesthesia (pg/ml)	24 hours after operation (pg/ml)
Control group (*n* = 50)	151.82 ± 32.11	219.05 ± 52.02^*∗*^
Research group (*n* = 50)	151.69 ± 32.03	175.03 ± 41.01^*∗*^
*t* value	0.020	4.699
*p* value	0.984	<0.01

Note: the symbol^*∗*^represents the comparison of 24 hours before and 24 hours after anesthesia induction in this group, *p* < 0.05.

**Table 4:** Comparison of cortisol levels before and 24 hours after anesthesia induction.

Group	Before induction of anesthesia (ng/ml)	24 hours after operation (ng/ml)
Control group (*n* = 50)	82.12 ± 18.39	174.19 ± 39.25^*∗*^
Research group (*n* = 50)	82.14 ± 18.44	129.23 ± 30.35*∗*
*t* value	0.005	6.408
*p* value	0.996	<0.01

Note: the symbol^*∗*^represents the comparison of 24 hours before and 24 hours after anesthesia induction in this group, *p* < 0.05.

**Table 5:** Comparison of the score of the SAS scale and the RSS scale during the recovery period of anesthesia.

Group	SAS scale (score)	RSS scale (score)
Control group (*n* = 50)	53.52 ± 4.12	3.24 ± 0.05
Research group (*n* = 50)	47.49 ± 1.09	5.18 ± 0.13
*t* value	10.005	98.489
*p* value	<0.01	<0.01

**Table 6:** Comparison of the recovery time of the bowel sound and the anal exhaust time after operation.

Group	Postoperative bowel sound recovery time (h)	Anal exhaust time (h)
Control group (*n* = 50)	57.23 ± 3.37	80.29 ± 2.64
Research group (*n* = 50)	38.18 ± 2.42	58.71 ± 1.15
*t* value	32.467	52.991
*p* value	<0.01	<0.01

**Table 7:** Comparison of the incidence of gastrointestinal adverse reactions 24 hours after operation.

Group	Nausea (case/%)	Vomiting (case/%)	Abdominal distension (case/%)	Incidence of gastrointestinal adverse reactions (case/%)
Control group (*n* = 50)	2/4.00	3/6.00	5/10.00	10/20.00
Research group (*n* = 50)	1/2.00	0/0.00	1/2.00	3/4.00
*t* value				4.640
*p* value				0.031

## Data Availability

The datasets used and analyzed during the current study are available from the corresponding author upon reasonable request.
